The article "circRNA circFAT1(e2) Elevates the Development of Non-Small-Cell Lung Cancer by Regulating miR-30e-5p and USP22" was published in 2021. Journal: Biomed Res Int.

# circRNA circFAT1(e2) Elevates the Development of Non-Small-Cell Lung Cancer by Regulating miR-30e-5p and USP22

**DOI:** 10.1155/2021/6653387

**Published:** 2021-04-02

**Authors:** Wenmin Dong, Huiqian Zhang, YanCheng Dai, Yi Zhou, Yun Luo, Cheng Zhao, Yiyuan Cao, Yuping Du, Ying Chen

**Affiliations:** ^1^Shanghai TCM-Integrated Hospital Affiliated to Shanghai University of Traditional Chinese Medicine, Shanghai 200082, China; ^2^Shanghai University of Traditional Chinese Medicine, Shanghai 201203, China

## Abstract

**Background:**

As a newly discovered regulatory RNA, circular RNA (circRNA) has become a hot spot in many tumor pieces of research. In recent years, it has been discovered that circRNAs have multiple biological effects in different stages of cancer. However, the expression pattern and mechanism of circFAT1(e2) in non-small-cell lung cancer (NSCLC) are still unclear.

**Methods:**

The expressions of circFAT1(e2) in NSCLC tissues and cell lines were studied. Functionally, CCK-8 and transwell experiments were performed in A549 and H1299. In addition, we also performed a dual-luciferase report analysis to clarify the mechanism of action of circFAT1(e2).

**Results:**

circFAT1(e2) was significantly upregulated in NSCLC tissues and cell lines. circFAT1(e2) gene knockdown could significantly inhibit the proliferation, migration, and invasion of NSCLC cells. Loss of function testing found that circFAT1(e2) functioned as an oncogene in NSCLC cells. In addition, circFAT1(e2) acted as a ceRNA to spongy miR-30e-5p, which led to the increase in USP22 and promoted cell growth.

**Conclusions:**

The circFAT1(e2)-miR-30e-5p-USP22 axis is a crucial part of the progression of NSCLC. This study suggests that circFAT1(e2) may be an important potential of prognostic prediction and treatment targets for NSCLC patients.

## 1. Introduction

The tumorigenesis of cancer is due to the abnormal changes of regulatory mechanisms in cells, resulting in uncontrolled growth and division [1]. However, the mechanisms underlying tumorigenesis remain unclear. circRNA is a novel type of ncRNAs (noncoding RNAs) and exists in both the cytoplasm and nucleus of eukaryotes [2]. It is characterized by a ring-shaped structure without free ends [3]. circRNA is produced through special types of alternative splicing [4]. With the deepening of research, the understanding of circRNA has been gradually enriched. The reverse splicing pathway of exons is the key mechanism involved in producing circRNAs [5]. Of note, emerging studies demonstrate circRNAs play important roles in regulating the development of cancers [6]. For example, studies have found that the downregulated expression of circRNA circ-Ccnb1 in breast cancer can interact with Bclaf1 in cancer cells through H2AX, resulting in the inhibition of uncontrolled division and growth of cancer cells [7]. Researchers also find that circITGA7 can inhibit the metastasis and proliferation of colorectal cancer cells by inhibiting the pathway of Ras signal and promoting the transcription of its downstream target gene ITGA7, thus playing its antitumor roles in colorectal cancer [8].

The article "circRNA circFAT1(e2) Elevates the Development of Non-Small-Cell Lung Cancer by Regulating miR-30e-5p and USP22" was published in 2021. Journal: Biomed Res Int.

According to the latest reports, among all kinds of cancers, lung cancer leads to the highest morbidity and mortality [9]. More than 2 million new cases are diagnosed as NSCLC, and 1.8 million deaths are caused by NSCLC per year [10]. NSCLC can be divided into two subtypes, small-cell lung cancer (SCLC) and non-small-cell lung cancer (NSCLC). NSCLC includes large-cell NSCLC, lung squamous cell carcinoma, and lung adenocarcinoma [11]. Clinically, NSCLC is diagnosed mainly by small biopsies and cytological specimens [12]. According to recent reports, there are significant differences in circRNA expression levels between NSCLC tissues and normal tissues. It suggests that they may be involved in different stages or pathways of cancer cell progression [13]. It is found that NSCLC lowly expressed circRNA-ITCH which could be used as a sponge of miR-7 and miR-214, reducing their expression levels, reducing the regulatory effect of miRNA on downstream target genes, resulting in downregulation of b-catenin, c-myc, and cyclinD1, and then inhibiting the activation of Wnt/b-catenin signal in NSCLC cells [14]. In addition, Luo et al. found that hsa_circ_0000064 expression increased in NSCLC tissues and cell lines, suggesting that this circRNA might be an oncogene. Gene knockout experiment showed that the proliferation, migration, and invasion of NSCLC cells were significantly inhibited, the cell cycle process was accelerated, and the number of apoptotic cells increased [15].

Previous studies have shown that circFAT1(e2) is a new circRNA derived from exon 2 of the FAT1 gene [16]. In PTC, circFAT1(e2) plays a carcinogenic effect by promoting cell invasion and metastasis and is a potential new target for PTC therapy [17]. It is found in gastric cancer (GC) that the overexpression of circFAT1(e2) inhibits the proliferation, migration, and invasion of GC cells and is related to the overall survival rate of GC patients [16]. Studies in osteosarcoma (OS) show that circFAT1(e2) plays a carcinogenic role in OS and suggest that the circFAT1(e2)/miR-181b/HK2 axis is a potential therapeutic target [18]. However, the function and mechanism of circFAT1(e2) related to NSCLC are still unclear.

In this study, we observed that circFAT1(e2) was highly expressed in NSCLC tissues compared with normal tissues. We found that the proliferation ability of NSCLC cells was significantly limited, and the ability to invade and metastasize was also significantly decreased after knockdown of circFAT1(e2) with siRNA. Using the luciferase reporter assay, it was found that circFAT1(e2) could reduce the activity of miR-30e-5p by acting as a sponge, which weakened the regulation of the downstream target gene USP22, and finally restricted the metastasis and growth of NSCLC cells. We could provide new targets and pathways to regulate the development of NSCLC, which had potential value as a target for screening and diagnosis of NSCLC.

The article "circRNA circFAT1(e2) Elevates the Development of Non-Small-Cell Lung Cancer by Regulating miR-30e-5p and USP22" was published in 2021. Journal: Biomed Res Int.

## 2. Materials and Methods

### 2.1. Patients and Tissue Samples

We collected paired NSCLC tissue and adjacent normal tissue from 5 patients who underwent surgical resection without any chemoradiotherapy at the Shanghai TCM-Integrated Hospital affiliated to Shanghai University of Traditional Chinese Medicine. We stored the resected tissues immediately in liquid nitrogen at -80°C for further RNA isolation. All experiments were approved by the Institutional Review Board, and all patients provided informed consent in writing prior to participation.

### 2.2. Cell Lines and Cell Culture

We collected the NSCLC cells (A549, H1299, and NCI-H1975) and normal cells (BEAS-2B) from the American Type Culture Collection. We then maintained the cells in RPMI-1640 and supplemented them with 100 U/mL penicillin, 100 *μ*g/ml streptomycin, and 10% fetal bovine serum (FBS). A humidified incubator with 5% carbon dioxide at 37°C was applied. The culture medium was changed every 3 days.

### 2.3. Cell Transfection

siRNA was purchased from GenePharma Co., Ltd. (Shanghai, China). The siRNA sequence was as follows: si-circFAT1(e2), GAGACAGATTCCCGACAGTTADTDT, and si-NC, UUCUCCGAACGUGUCACGUTT. When the cells reached 80% confluence, the cells used for transfection were plated in a 6-well plate. According to the manufacturer's protocol, all transfections were performed using Lipofectamine 2000 (Invitrogen, Carlsbad, CA, USA). Cells were harvested 48 hours after transfection for subsequent experiments.

### 2.4. RNA Extraction and qRT-PCR

The TRIzol reagent was used to extract total RNA from NSCLC cells. The PrimeScript RT reagent kit was used to reverse-transcribe the isolated RNA (1 *μ*g) into cDNA. qRT-PCR was performed using the StepOne™ Real-Time PCR System and the SYBR® Green Mixture. Relative data were normalized to GAPDH.

### 2.5. CCK-8 Assay

The Cell Counting Kit-8 (CCK-8) was used to examine the proliferation ability of NSCLC cells (A549, H1299). By the manufacturer's instructions, at a specific time, we added CCK-8 (10 *μ*L per well) to the cells after transfection and incubated them for two hours before measuring the absorbance at 450 nm.

The article "circRNA circFAT1(e2) Elevates the Development of Non-Small-Cell Lung Cancer by Regulating miR-30e-5p and USP22" was published in 2021. Journal: Biomed Res Int.

### 2.6. Transwell Migration and Invasion Assay

After 12 hours of transfection, we seeded the cells (1 × 10^5^ cells/well) into the upper transwell chamber for the migration assay, or cells were preapplied with 70 *μ*L diluted Matrigel for the invasion assay, with 100 *μ*L of RPMI-1640 medium containing 1% FBS. After 48 hours, we wiped the cells on the upper surface with a cotton swab, fixed them with methanol, and then stained them with 10 *μ*g/mL DAPI (Solarbio, Beijing, China).

### 2.7. Public Database

The GSE9188 database [19] (https://www.ncbi.nlm.nih.gov/geo/query/acc.cgi) contains 5 subdatasets, and the GEO2R online network tool (https://www.ncbi.nlm.nih.gov/geo/geo2r/?acc=GSE9188) allows users to compare different gene expression data of two or more sets of samples. We use GEO2R to analyze gene expression levels. Through bioinformatics tools circBase (http://www.circbase.org/) and starBase 2.0 (http://starbase.sysu.edu.cn/starbase2/index.php), we determined the downstream of the circFAT1(e2) target gene.

### 2.8. Dual-Luciferase Reporter Assay

USP22 mRNA wild type (USP22-3UTR-wt) or circFAT1(e2) wild type (circFAT1(e2)-wt) with potential miR-30e-5p binding sites and mutant without miR-30e-5p binding sites (USP22-3UTR-mut, circFAT1(e2)-mut) were constructed for the dual-luciferase reporter assay. Then, we amplified and cloned them into the luciferase reporter vector psi-CHECK-2. We cotransfected HEK293T cells with luciferase plasmids and miR-30e-5p or control. The Dual-Luciferase Reporter Assay System was employed based on the Renilla luciferase activity.

### 2.9. Statistical Analysis

We performed Student's *t*-test or one-way ANOVA to test the differences between groups. Each experiment was repeated at least three times. Data were presented as mean ± SD (standard deviation). The *P* value less than 0.05 was considered statistically significant. The SPSS software was used to perform all the statistical analyses, and the GraphPad Prism software was used to graph.

## 3. Results

### 3.1. circFAT1(e2) Was Probably Overexpressed in the NSCLC Tissue and Cells

In this study, we aimed to explore the potential functions of circFAT1(e2) in NSCLC. In the 5 clinical NSCLC tissues, circFAT1(e2) expression was significantly overexpressed (Figure 1(a)), and the results were similar in NSCLC cells (Figure 1(b)). It suggested that circFAT1(e2) was probably overexpressed in NSCLC tissues and cells.

### 3.2. circFAT1(e2) Knockdown Repressed the Proliferation and Metastasis of NSCLC Cells

Loss-of-function experiments were performed using siRNA targeting circFAT1(e2) in NSCLC cells (A549, H1299) (Figure 2(a)). The CCK-8 assay was carried out to investigate the inhibition of circFAT1(e2) knockdown on cell proliferation (Figure 2(b)). The transwell assay was carried out and found that circFAT1(e2) knockdown inhibited the invasion and migration of NSCLC cells compared to the control group (Figure 2(c)). These results indicated that circFAT1(e2) knockdown represses the metastasis and proliferation of NSCLC cells.

The article "circRNA circFAT1(e2) Elevates the Development of Non-Small-Cell Lung Cancer by Regulating miR-30e-5p and USP22" was published in 2021. Journal: Biomed Res Int.

### 3.3. circFAT1(e2) Targeted miR-30e-5p as a miRNA Sponge

Research shows that circRNAs can target miRNAs by acting as miRNA sponges and binding with the RNA-binding protein (RBP) to exert their function. Results from this study found that miR-30e-5p had complementary binding sites with the circFAT1(e2). The luciferase activity demonstrated the interaction between the molecular binding of circFAT1(e2) and miR-30e-5p (Figure 3(a)). Results also found that miR-30e-5p was highly expressed in the circFAT1(e2) knockdown transfection in the NSCLC cells (Figure 3(b)). However, we found that overexpression of miR-30e-5p remarkably suppresses the expression level of circFAT1(e2) in both A549 and H1299 cells (Figure 3(c)). The results suggest that circFAT1(e2) serves as a miRNA sponge for miR-30e-5p.

### 3.4. USP22 Served as the Functional Protein of circFAT1(e2)/miR-30e-5p

Further experiments were aimed at investigating the downstream target of circFAT1(e2) and miR-30e-5p. Previous reports indicated that USP22 was a potential target of miR-30e-5p [20, 21]. In this study, the dual-luciferase assay also validated the molecular binding between miR-30e-5p and USP22 mRNA (Figure 4(a)). The expression of USP22 in NSCLC tissues was higher than that in normal tissues using the GSE9188 database (Figure 4(b)). We also found that overexpression of miR-30e-5p and knockdown of circFAT1(e2) significantly reduced the mRNA levels of USP22 (Figures 4(c) and 4(d)). RT-PCR illustrated that USP22 mRNA expression was increased in the miR-30e-5p silencing group, which was recovered by circFAT1(e2) siRNA (Figure 4(e)). These results demonstrate that USP22 acts as the functional protein of circFAT1(e2)/miR-30e-5p.

## 4. Discussion

NSCLC, as the deadliest cancer in the world, has received extensive attention [22]. Although many countries have begun to pay attention to and take measures to restrict smoking to prevent NSCLC, the incidence and mortality of NSCLC are still increasing [23]. Understanding the molecular pathogenesis of NSCLC is helpful to improve the life quality and prolong the survival time of patients [24]. As a large number of important substances are involved in cell regulation, circRNA is playing more and more important roles in the diagnosis and treatment of cancer [25]. Our study found that the expression level of circFAT1(e2) in normal tissues is lower than that in NSCLC tissues. Using a series of experiments, it was found that circFAT1(e2) could decrease the expression level of miR-30e-5p, which in turn inhibited miR-30e-5p on the regulation of the downstream target gene USP22. This study demonstrated that knockdown of circFAT1(e2) decreased the ability of NSCLC cells to proliferate, invade, and metastasize.

The article "circRNA circFAT1(e2) Elevates the Development of Non-Small-Cell Lung Cancer by Regulating miR-30e-5p and USP22" was published in 2021. Journal: Biomed Res Int.

A large number of noncoding RNAs such as miRNAs, lncRNAs, and circRNAs existed in cells, [26]. Current studies have found that circRNAs may be used as a ceRNA to competitively bind to miRNA binding sites, thus interfering with the activity of miRNAs to regulate downstream target genes [27]. For example, ciRS-7 can affect the binding activity of miR-7 [28]. In addition, studies have found that CIRC_0067934 directly inhibits the interaction between mRNA 3′-UTR of FZD5 and miR-1324 and activates the FZD5/Wnt/*β*-catenin signal pathway to promote the proliferation, invasion, and migration of hepatocellular carcinoma cells [29]. The circFAT1(e2) is derived from exon 2 of the FAT1 gene. Studies in gastric cancer cells have shown that overexpressed circFAT1(e2) inhibits the proliferation, migration, and invasion of gastric cancer cells by targeting binding to miR-548g and releasing RUNX1 [16]. In contrast, our results in NSCLC show that circFAT1(e2) knockdown can inhibit the growth of NSCLC cells. The highly expressed circFAT1(e2) decreases the activity of miR-30e-5p through competitively binding with miR-30e-5p, thus promoting the invasive ability and growth of NSCLC cells.

Ubiquitin-specific protease 22 (USP22), as a part of the mammalian SAGA complex, can affect histone modifications by deubiquitination of H2A and H2B, which is one of the key regulators of the cell cycle. Studies have shown that overexpression of USP22 can enhance the inhibitory effect of cell cycle inhibitors such as p21 and enhance the proliferation of tumor cells, thus promoting the occurrence and development of tumors [30]. By knocking out circFAT1(e2), we found that the ability of cells to proliferate, invade, and metastasize was significantly inhibited. Luciferase report experiment showed that overexpressed circFAT1(e2) could sponge miR-30e-5p and reduce the expression level of this miRNA, thus weakening the regulation of miR-30e-5p on the downstream target gene USP22 and increasing the expression of USP22.

In addition, this study has some limitations. First of all, although the expression level of circFAT1(e2) was detected in a small sample size of NSCLC samples, a larger sample size should be used to further verify the correlation between the expression of circFAT1(e2), miR-30e-5p, and USP22 and clinical parameters. Second, the findings of this study were derived from in vitro analysis. Therefore, *in vivo* analysis should be performed to further verify our findings.

The article "circRNA circFAT1(e2) Elevates the Development of Non-Small-Cell Lung Cancer by Regulating miR-30e-5p and USP22" was published in 2021. Journal: Biomed Res Int.

In conclusion, the present study for the first time demonstrated that circFAT1(e2) acted as an oncogene in NSCLC, and circFAT1(e2) promoted NSCLC cell proliferation, migration, and invasion. Using a series of experiments, we found that circFAT1(e2) knockdown decreased the expression level of USP22 through sponging miR-30e-5p. Our study indicated that circFAT1(e2) might be a potential biomarker of NSCLC and provided a variety of options for screening, diagnosis, and treatment of NSCLC.

## Figures and Tables

**Figure 1:** In the NSCLC tissue and cells, circFAT1(e2) was overexpressed. (a) As shown by qRT-PCR analysis, the relative expression levels of circFAT1(e2) (*n* = 5) in the matched noncancerous tissues and NSCLC tissues. (b) As shown by qRT-PCR, circFAT1(e2) expression in three CRC cell lines was also higher than that in the normal cell line BEAS-2B. ^∗^*P* < 0.05, ^∗∗^*P* < 0.01.

**Figure 2:** circFAT1(e2) knockdown repressed NSCLC cells' metastasis and proliferation. (a) To knock down circFAT1(e2) level, siRNA which specifically targeted the circFAT1(e2) (si-circFAT1(e2)) were transfected into NSCLC cells. (b) That circFAT1(e2) downexpression inhibited NSCLC cell proliferation was demonstrated by the CCK-8 assay. (c) That knockdown of circFAT1(e2) decreased cell invasion and migration was indicated by transwell assays. ^∗^*P* < 0.05.

**Figure 3:** circFAT1(e2) targeted miR-30e-5p as a miRNA sponge. (a) The dual-luciferase reporter assays indicated that luciferase activity was decreased in HEK 293T cells after cotransfecting with circFAT1(e2)-wt and miR-30e-5p. (b) In NSCLC cells that knocked down circFAT1(e2), the expression of miR-30e-5p was higher. (c) In miR-30e-5p overexpression cells, circFAT1(e2) expression decreased. ^∗^*P* < 0.05.

**Figure 4:** USP22 served as the functional protein of circFAT1(e2)/miR-30e-5p. (a) The relative fluorescence intensity was confirmed by the luciferase reporter assay when the cotransfection between USP22 3′-UTR wild-type or mutant and miR-30e-5p or control happened. (b) There was difference between the expression of USP22 in normal tissues and that in NSCLC tissues. (c) After overexpression of miR-30e-5p, USP22 mRNA levels decreased. (d) USP22 mRNA level decreased after knockdown of circFAT1(e2) in A549 and H1299 cells. (e) USP22 mRNA expression can be increased by the miR-30e-5p inhibitor which can also resist the reduction of USP22 mRNA caused by circFAT1(e2) knockdown. ^∗^*P* < 0.05, ^∗∗^*P* < 0.01, and ^∗∗∗^*P* < 0.001.

The article "circRNA circFAT1(e2) Elevates the Development of Non-Small-Cell Lung Cancer by Regulating miR-30e-5p and USP22" was published in 2021. Journal: Biomed Res Int.

## Data Availability

The datasets used and/or analyzed during the current study are available from the corresponding author on reasonable request.

## Abbreviations

ncRNA: Noncoding RNA
circRNA: Circular RNA
NSCLC: Non-small-cell lung cancer
ncRNAs: Noncoding RNAs
SCLC: Small-cell lung cancer
FBS: Fetal bovine serum
CCK-8: Cell Counting Kit-8
RBP: RNA-binding protein
USP22: Ubiquitin-specific protease 22.
